RETRACTED

# To Analyze the Mechanism of SalB Regulating SIRT1 to Inhibit NLRP3 and Its Ameliorative Effect on Tubulogastric Junction Tumor Lesions Complicated with Myocardial Injury

**DOI:** 10.1155/2022/6560693

**Published:** 2022-10-14

**Authors:** Guo-Ping Wang, Zheng Guo

**Affiliations:** ^1^Changzhi People's Hospital of Shanxi Medical University, Changzhi, Shanxi 046000, China; ^2^Department of Anesthesiology, Second Hospital of Shanxi Medical University, Taiyuan, Shanxi 03001, China

## Abstract

The objective of this research is to investigate the mediating impact of salvianolic acid B (SalB) on SIRT1 signaling pathway and the mechanism by which it inhibits Nod-like receptor protein 3 (NLRP3), as well as to examine how SalB affects myocardial injury brought on by tumor lesions at the junction of the tube and the stomach. Through the establishment of the integration of a stomach tube tumor lesion rats combined with the experimental rat model, this study establishes the normal group, model group, and different SalB dose groups. For each group of cells, cell activity and cell apoptosis were determined and compared using colorimetry and enzyme-linked immunosorbent method about lactate dehydrogenase (LDH). Interleukin-1 beta levels are measured. DCFH-DA fluorescent probe was applied to identify intracellular “reactive oxygen species” (ROS). “Western blot” was used to determine NLRP3, caspase-1, and apoptosis-related spotted protein (ASC) in each group of cells. And SIRT1 signaling pathway related to SIRT1, phosphorylated AMP protein-activated kinase *α* (P-AMPK *α*), AMP protein-activated kinase *α* (AMPK*α*), and “peroxisome-proliferator-activated receptor *γ* coactivator 1*α* (PGC-1*α*) protein expression” are used. According to the final findings, SalB mediated the SIRT1 signaling pathway and had a beneficial impact on the upregulation of SIRT1, P-AMPK/AMPK, and PGC-1 protein expressions. SalB positively affects the downregulation of NLRP3 inflammasome-related proteins. Caspase-1 and ASC protein expression suggesting that SalB may inhibit the activation of NLRP3 inflammasome induced by oxidative stress by activating SIRT1/AMPK/PGC-1*α* signaling pathway. This plays an antimyocardial injury effect.

## 1. Introduction

Myocardial ischemic injury is a cardiac pathological state caused by coronary artery obstruction. Reduced myocardial perfusion may eventually result in ischemic cardiomyopathy and heart failure because of disproportionate supply and demand of oxygen [1]. According to studies [2, 3], myocardial ischemia injury is caused by aseptic inflammation, which is intervened by the Nod-like receptor protein 3 (NLRP3) inflammasome. One of Salvia miltiorrhiza's main water-soluble components is called SalB. Studies [4–6] reveal that SalB can prevent myocardial ischemia through its anti-inflammatory and antioxidant properties. Salvianolic acid B has a myocardial ischemia effect which is associated to its inhibition of NLRP3 inflammasome activation.

RETRACTED

Silencing information regulator 1(SIRT1) is considered to be an important protective molecule of the heart. As a deacetylase is dependent on nicotinamide adenine dinucleotide (NAD+), SIRT1 can exert antioxidant, apoptosis reduction, anti-inflammatory, and energy metabolism regulation effects through deacetylated related factors [7]. Previous studies [8] have found that SIRT1 agonist may reduce the activation of NLRP3 inflammasome. It is not clear whether salvianolic acid B inhibition of NLRP3 inflammasome activation is related to regulation of SIRT1 signaling pathway. In addition, for the integration of a stomach tube in clinical tumor lesions in patients with gastrointestinal surgery intervening treatment, surgical intervention can improve the symptoms of such patients, but the patients are likely to be effected by surgical injury and myocardial injury. This is also a heart surgery after one of the most important attributable mortality risk [9]. Based on this, the current work established a rat model of an esophagogastric junction tumor and performed tests to determine whether SalB inhibits NLRP3 inflammasome activation by upregulating SIRT. It also observes the effect on tubulogastric junction tumor lesions combined with myocardial injury. The findings are listed below.

## 2. Instruments and Material

### 2.1. Experimental Animals

Every rat model included in this study was purchased from Beijing Institute of Life Sciences including 72 SPF healthy rats aged 8-10 weeks, with a body weight of (215.50 ± 10.50) g. Experimental Animal Production License Number is SCXK (Beijing) 2018-0008, and Animal Quality Certificate Number is 2021061703. Temperature during the experiment was between 22 and 24°C and relative humidity ranged from 50 to 70 percent. All rats were fed strictly in accordance with animal feeding guidelines.

### 2.2. Cell Lines

“The Cell Center of the Institute of Basic Medical Sciences” of Chinese Academy of Medical Sciences provided human esophageal cancer Eca109 cells. Nanjing KGI Biotechnology Co., Ltd. provided the cardiac muscle cell line H9c2. H9c2 cardiomyocytes were refined and cultured in a high glucose medium with 10% fetal bovine serum and kept at 37°C with 5% CO_2_ in a cell incubator. Every two days, the cells were subcultured once.

### 2.3. Drugs and Reagents

SalB was purchased from “Shanghai Yuanye Biotechnology Co., Ltd.” with Batch Number: B20261. 3% hydrogen peroxide (H_2_O_2_) was provided by Sigma Company, USA, having Article No. STBH9407. EX527 (SIRT1-specific inhibitor), MCE Inc., HY-15452, and DMEM Culture Medium were purchased from “Nanjing KGI Biotechnology Co., Ltd.” The Batch Number was 20200923. Fetal bovine serum was provided by BI Biotechnology Israel with Article No. 04-001-1ACS. Thiazolyl blue (MTT) was purchased from “Guangzhou Saiguo Biotechnology Co., Ltd.” Batch Number was EZ2811A179. Rat IL-1*β* Detection Kit was purchased from “Hangzhou Lianke Biotechnology Co. Ltd.” Batch Number was A301B91044. Lactate dehydrogenase (LDH) detection kit (Batch No. 121719200413), Hoechst staining kit (Batch No. 122419200512), and reactive oxygen species (ROS) detection kit (Batch No. 011520200504) were purchased from “Shanghai Biyuntian Biotechnology Co., Ltd.” *β*-actin antibody was provided by “Shanghai Bowan Biotechnology Co., Ltd.” having Article. No. AB0035. NLRP3 antibody (article No. BS-10021R), cysteine aspase-1 antibody (article No. BS-10442R), and apoptosis related spotted protein (ASC) antibody (article No. BS-6741R) were purchased from “Beijing Boaosen Biotechnology Co., Ltd.” SIRT1 antibody was purchased from “CST Company, USA.” Article No. was D1D7. Phosphorylated AMP protein-activated kinase *α* (P-AMPK *α*) antibody (AP1171), AMP protein-activated kinase *α* (AMPK*α*) antibody (A17290), and peroxisome-proliferator-activated receptor *γ* coactivator 1*α* (PGC-1*α*) antibody (PGC-1*α*) A11971) were all purchased from “Wuhan AIbotec Biotechnology Co., Ltd.”

RETRACTED

### 2.4. Main Instruments

This includes Synergy2 Multifunctional Microplate Tester, BioTek, USA; Allegra 64R superspeed refrigerated centrifuge, Beckman Company, USA; Discovery.V20 Fluorescence inverted microscope, ZEISS, Germany; and Model 164-5050 electrophoresis apparatus and GelDoc-2000 Gel Imager, Bio-Rad Company, USA.

### 2.5. Cell Grouping and Treatment

Excluding 12 rats in the normal group, the left over 60 rats were prepared by referring to the methods of literature, etc. [10]. Human Eca109 cells were cultured in vitro and routinely digested by trypsin for passage. After centrifugation, logarithmic growth phase cells were collected, and the density of cell was increased to 1 × 10^7^ cells per milliliter by suspending the cells in D-Hanks solution. The rats' axillae were then subcutaneously injected with 0.5 mL of cell solution. When the tumor volume is 100 mm^3^, the modeling is successful. H9c2 cells at the logarithmic development stage were inoculated in 96-well and 6-well plates for 24 hours, respectively, after successful modeling. Cells were separated into model group and SalB group with various dosages in accordance with the experimental requirements. The normal group cells were cultured in the incubator at 37°C for 48 hours and then refined and cultured in DMEM incomplete medium for 4 h. After 48 hours growth in the cell incubator, cells in the model group were stimulated with 600 *μ*mol/L H_2_O_2_ for 4 hours. After the cells in the SalB group were grown in cell incubator for 24 hours, salvianolic acid B (5, 10, 20 *μ*mol/L) was added to incubate for 24 hours, and then 600 *μ*mol/L H_2_O_2_ was added for 4 hours.

RETRACTED

### 2.6. Use of MTT Assay for the Detection of Cell Viability

H9c2 cells at logarithmic growth stage were taken. Cells in the 96-well plate were grouped according to 1.5 content and treated with corresponding drugs. Following incubation at 37°C and 5% CO_2_, the supernatant was removed, and each well received 200 L of DMEM high sugar incomplete medium before receiving 20 L of MTT solution (5 mg/mL). 4 hours were spent incubating at 37°C, after which the supernatant was absorbed and removed. To avoid light, each well then received 150 L of DMSO solution, which was then gently stirred and shaken for 10 min to dissolve the dirty crystals. At 570 nm, the optical density (OD) of each hole was determined.

### 2.7. Hoechst Staining to Detect Cell Apoptosis

The cell slides sterilized by 75% alcohol were placed in the 6-well plate. H9c2 cells at logarithmic growth stage were taken. The cells in the 6-well plate were grouped according to 1.5 and treated with corresponding drugs. The supernatant was removed after being incubated at 37°C and 5% CO_2_ and washed 3 times in sterile PBS and once in DMEM incomplete high sugar medium. Each well received 1 mL of fixative, which was then added, incubated overnight at 4°C, and rinsed three times for three minutes each in sterile PBS. 0.5 mL Hoechst staining solution was added to each well for staining for 5 min. The staining solution was then removed and washed with PBS twice for 3 min each. The supernatant was vacuumed and photographed under a fluorescence microscope.

### 2.8. Detection of LDH Release by Colorimetry

H9c2 cells in the logarithmic growth phase were immunized into 96-well plates, classified according to 1.5, and given the appropriate and corresponding drug treatments. After H_2_O_2_ stimulation, the cell supernatant was gathered and centrifuged at 2000 rpm for 10 minutes with a 10 cm radius to remove the precipitate. The LDH working reagent was coincubated with the treated cell supernatant for 30 min before being transferred to a fresh 96-well plate. Using a microplate reader, OD values were measured at 450 nm.

### 2.9. ROS Release and Detection by DCFH-DA Method

The level of the ROS was assessed using the DCFA-DA fluorescent probe. By diluting dCFH-DA with serum-free cell culture medium, the final concentration of DCFH-DA was 10 mol/L. Each group's H9c2 cells were gathered, suspended in diluted DCFH-DA, and incubated for 20 min at 37°C. The fluorescence intensity was analyzed at 488 nm excitation wavelength and 525 nm emission wavelengths using a microplate reader.

RETRACTED

### 2.10. Detection of Interleukin-1*β* (IL-1*β*) by ELISA

H9c2 cells in logarithmic growth phase were immunized into 6-well plates, and cells were grouped according to 1.5 and treated with corresponding drugs. After H_2_O_2_ stimulation, cell supernatant was collected and centrifuged with a centrifugation radius of 10 cm and 2000 r/min for 10 min to remove the precipitate. The amount of IL-1 in the cell supernatant was measured strictly in accordance with the ELISA kit's instructions.

### 2.11. Use of Western Blot for the Detection of Expressions of NLRP3 Inflammasome and SIRT1 Signaling Pathway-Related Proteins

After cell grouping and treatment according to 1.5, H9c2 cells in each group were lysed in RIPA lysis buffer containing phosphatase inhibitors. The supernatant was removed using a centrifuge with a 10 cm radius and centrifuged for 15 minutes at 12 000 rpm to determine the total protein content using a BCA kit. 30 *μ*g protein of each group was separated by SDS-PAGE and shifted to PVDF membrane. 5% skimmed milk powder was used for sealing at room temperature for 1 h, and corresponding primary antibody (1 : 1000) was added and incubated overnight at 4°C. Second antibody (1 : 5000) was added and incubated at room temperature for 2 h. The ECL chemiluminescence method was used to detect the target band. The ratio of the gray value of the target band to the internal reference band (*β*-actin) was used to measure the protein expression level of the target band.

### 2.12. Statistical Treatment

Data analysis was executed using statistical software named SPSS 22.0, and measurement data were reported as mean ± standard deviation. LSD test was performed for pairwise comparison, while one-way ANOVA was utilized to compare data from various groups. The difference was of statistical significance when *P* > 0.05.

## 3. Discussion and Results

### 3.1. Effect of SalB on H_2_O_2_-Induced Injury of H9c2 Cells

In comparison to the normal group, there was significant decrease in the cell viability of the model group, whereas a significant rise was observed in the LDH activity of the model group (all *P* < 0.05). Comparison between SalB groups with different concentrations and model group showed that SalB could improve cell viability in a dose-dependent manner and reduce LDH activity with statistical significance (*P* < 0.05). It suggests that SalB could alleviate oxidative stress damage of H9c2 cells caused by H_2_O_2_ as shown in Figures 1 and 2.

RETRACTED

### 3.2. SalB Effect on H_2_O_2_-Induced Apoptosis of H9c2 Cells

By observing the status of cells in each group under fluorescence microscope, it could be seen that the nuclei of the normal group cells demonstrated uniform fluorescence and low fluorescence intensity. Comparison between the model group and the normal group showed that the model group cells had nuclear rupture. The color was white, the nucleus was dense and stained, and the degree of apoptosis was considerably increased (*P* < 0.05). Comparison between the SalB intervention group and model group after treatment showed that the number of cell chromatin pyknosis and white nuclei decreased significantly. The degree of cell apoptosis also decreased significantly (*P* < 0.05). These findings suggested that SalB could inhibit the apoptosis of H9c2 cells induced by H_2_O_2_ oxidative stress, see Figure 3 for details.

### 3.3. SalB Effect on ROS in H_2_O_2_-Induced H9c2 Cells

The ROS content in the model group showed a greater increase than the normal group (*P* < 0.05). When compared to the model group, the release of intracellular ROS showed a major decrease after SalB intervention with different concentrations (*P* < 0.05). This suggests that SalB can reduce the generation of intracellular ROS induced by H_2_O_2_ oxidative stress in H9c2 cells as illustrated in Figure 4.

### 3.4. SalB Effect on Secretion of IL-1*β* in H9c2 Cells Induced by H_2_O_2_

The expression of IL-1*β* in supernatant of the model group was greatly increased than the normal group (*P* < 0.05). Compared with the model group, the content of IL-1*β* in supernatant of cells was significantly decreased after treatment with 20 *μ*mol/L SalB (*P* < 0.05). It was suggested that H_2_O_2_-induced oxidative stress could lead to massive release of proinflammatory cytokine IL-1*β* in H9c2 cells, and SalB intervention could effectively inhibit the release of IL-1*β* in H9c2 cells, as illustrated in Figure 5.

### 3.5. SalB Effect on NLRP3 Inflammatory Body Protein Expression in H_2_O_2_-Induced H9c2 Cells

NLRP3, caspase-1, and ASC protein expressions in the model group were higher than those in the normal group (*P* < 0.05). In comparison to the model group, SalB could dose-dependently downregulate NLRP3, caspase-1, and ASC protein expressions in H9c2 cells (all *P* < 0.05). This recommended that SalB could slow down the activation of NLRP3 inflammasome induced by H_2_O_2_ oxidative stress, as shown in Figure 6.

### 3.6. SalB Effect on SIRT1-Related Protein Expression in H_2_O_2_-Induced H9c2 Cells

SIRT1, P-AMPK *α*/AMPK*α*, and PGC-1*α* proteins in the model group showed a major decrease than the normal group (*P* < 0.05). In comparison to the model group, SIRT1, P-AMPK *α*/AMPK*α*, and PGC-1*α* proteins increased significantly after SalB intervention (*P* < 0.05). SalB's protective effect on cardiomyocytes may be related to SIRT1/AMPK/PGC-1*α* signaling pathway, as shown in Figure 7.

RETRACTED

## 4. Conclusion

Previous studies on patients with clinical myocardial injury have found that activation of “innate immune system” and exacerbation of “inflammatory response” are vital mechanisms of the pathological process of acute myocardial injury. Aseptic inflammation induced by activation of NLRP3 inflammasome performs a key function in ischemic injury. NLRP3 inflammasome, as a key component of innate immunity, is mainly composed of “Nod-like receptor protein 3 (NLRP3), apoptosis-associated spotted protein (ASC) and precursors of Caspase-1.” When the body is stimulated by external stimuli, NLRP3 inflammasome assembly is activated. The activated caspase-1 further lyses pro-IL-18 and pro-IL-1*β* forming mature IL-18 and IL-1*β* and inducing inflammatory responses [11, 12].

SalB is a water-soluble component that can be extracted from Salvia miltiorrhiza. Previous studies have shown that this substance can remove a large number of ROS produced in the process of oxidative stress in the body. The reduction of ROS content has a positive effect on alleviating the degree of myocardial ischemia injury and improving the activity of myocardial cells [13]. The finding and outcomes of the study exhibited that in comparison to normal cells, the viability of H9c2 cells induced by H_2_O_2_ was significantly decreased, and the apoptosis rate and LDH release amount in cell supernatant were significantly increased. However, after SalB intervention, the cell viability of each dose group increased significantly, and the degree of apoptosis and the release amount of LDH decreased significantly. It suggested that SalB intervention has a certain protective effect on myocardial cells affected by oxidative stress and can improve the degree of injury.

Much research is conducted on the activation mechanism of NLRP3 inflammasome [14, 15], suggesting that the activation mechanism is related to potassium ion outflow, release of trypsin from lysosomes, and production of ROS. The production of intracellular ROS is a key factor leading to activation of NLRP3 inflammasome. At same time, in the pathological process of myocardial ischemic injury, the generation and accumulation of oxygen free radicals in the body are an important influencing mechanism of myocardial ischemic injury [16]. The results of this study suggested that H9c2 cells were significantly overexpressed in NLRP3, ASC, and caspase-1 proteins related to NLRP3 inflammasome activation after H_2_O_2_ stimulation. And the level of IL-1*β* downstream of NLRP3 inflammasome was significantly increased. SalB inhibits this phenomenon suggesting that SalB can protect H9c2 cells from H_2_O_2_-induced cell damage by inhibiting oxidative stress and NLRP3 inflammatory body activation.

RETRACTED

Silencing information regulator 1 (SIRT1) is a homologous protein with the highest homology of yeast Sir2, which can play a protective role in myocardium through various ways such as antioxidant, anti-inflammatory, inhibition of apoptosis, and maintenance of energy metabolism. It plays an important role in the occurrence of diseases like myocardial ischemia, myocardial hypertrophy, and diabetic cardiomyopathy [17]. The findings revealed that SIRT1 and its related p-AMPK*α*/AMPK*α* and PGC-1*α* protein expressions were significantly downregulated after H_2_O_2_ oxidative stress, suggesting that both SIRT1 downregulation and NLRP3 inflammatory body activation may be involved in oxidative stress-induced cell damage. Salvianolic acid B pretreatment could significantly promote the expression of SIRT1, P-AMPK *α*/AMPK*α*, and PGC-1*α*. It is speculated that salvianolic acid B may improve the energy metabolism disorder during myocardial ischemia by upregulating SIRT1 and inhibit the activation of NLRP3 inflammasome induced by ROS during myocardial ischemia.

To sum up, SalB can open joint merger integration of a gastric tumor lesions myocardial injury caused by myocardial enzymes and the release of inflammatory cytokines and reduce tissue necrosis and inflammatory cell exudation. Its mechanism may be through increased clearing oxygen free radical that inhibits the increase of NLRP3, thus reducing the activation of downstream IL-1 beta to achieve the purpose of protection of ischemic myocardium. However, whether SalB can inhibit NLRP3 activation by protecting lysosome and its myocardial protection effect in patients with tumor-related lesions at the tubular gastric junction needs to be further studied in the future.

## Figures and Tables

**Figure 1:** LDH activity comparison.

**Figure 2:** Comparison of cell viability. Note: compared with the normal group, ^##^*P* < 0.05; compared with the model group, ^∗∗^*P* < 0.05.

**Figure 3:** Comparison of relative apoptosis. Note: comparison with the normal group, ^##^*P* < 0.05; comparison with the model group, ^∗∗^*P* < 0.05.

**Figure 4:** Comparison of ROS content. Note: comparison with the normal group, ^##^*P* < 0.05; comparison with the model group, ^∗∗^*P* < 0.05.

RETRACTED

**Figure 5:** Comparison of IL-1*β* expression. Note: comparison with the normal group, ^##^*P* < 0.05; comparison with the model group, ^∗∗^*P* < 0.05.

**Figure 6:** Comparison of NLRP3, caspase-1, and ASC protein expressions.

**Figure 7:** Comparison of SIRT1, P-AMPK *α*/AMPK*α*, and PGC-1*α* protein expressions. Note: comparison with the normal group, ^##^*P* < 0.05; comparison with the model group, ^∗∗^*P* < 0.05.

## Data Availability

The dataset used in this paper are available from the corresponding author upon request.
